# A Blockchain-Based Verifiable User Data Access Control Policy for Secured Cloud Data Storage

**DOI:** 10.1155/2022/2254411

**Published:** 2022-04-27

**Authors:** Xinlong LI

**Affiliations:** School of Computer Science, Hunan Institute of Technology, Hengyang 421002, China

## Abstract

Adding the adequate level of security of information systems dealing with sensitive data, privacy, or defense systems involves some form of access control. The audits performed are dealing with the determination of the allowed activities of the legal users, when attempting to access resources of the system. Usually, full access is provided after the user has been successfully authenticated through an authentication mechanism (e.g., password), while the corresponding authorization control is based on the confidentiality level of the respective resources and the authorization level assigned to each user. A very important diversification occurring in modern digital technologies is related to the identification based on blockchain technology, which is presented as a public, distributed data series, unable to modify its history and grouped in time-numbered blocks. In this work, a blockchain-based verifiable user data access control policy for secured cloud data storage is suggested for a version associated with big data in health care. It is an innovative system of applying classified access policies to secure resources in the cloud, which operates based on blockchain technology. System evaluation is carried out by studying a case in its resilience to Eclipse attack under different malicious user capabilities for routing table poisoning.

## 1. Introduction

Cloud data access control requires cooperation between processing sectors and at the same time protected and managed as a computational collaborative environment consisting of computational units under the management of distributed access control [1]. An access control state is said to be secure if no permission for access can lead to an unauthorized person. Blockchain [2] is a transparent, verifiable, permanent transactions management system operating and distributed in peer networks, offering and maintaining a robust mechanism of consensus, which, unlike the usual procedures, does not base its credibility and solvency on some reliable third entity.

In public blockchains, anyone interested can participate in the network, as access to their data is open by reading the chain and verifying the blocks, thus creating transparency in the information. This achieves the secure decentralization of the system since the members do not need to trust each other. On the other hand, there are many cases of applications where transactions or assets do not have to be disclosed or accessible to all, but by selected participants. Such transactions may be between competitors, medical history, transportation of goods, etc. [3]. That is the main reason why private blockchains were created. They are useful in cases where the integrity of the trace is not the most important prerequisite, and there is a need to standardize the exchange of information in a secure way between partners.

Combining the cloud and the blockchain can result in a verifiable [1, 4], permanent, and unmodified file in terms of data sharing between a private chain, eliminating the primary issue of supervision by allowing anybody permitted to join the network to observe and evaluate the activities transparently. In the event that something goes wrong with the processes (e.g., information leaks), blockchain makes it fairly straightforward to find the weak node [5]. Furthermore, the existence of a central service for storing and processing authentication information is not required for blockchain.

This capability is further strengthened by the blockchain's smart contracts [6]. They seek to provide security above and beyond contract law as well as to lower the additional transaction costs involved with the award and implementation of intermediate contracts. Furthermore, all users of this network can see blockchain-based contracts. This feature improves transaction transparency and dependability in complex contexts by intelligently automating the approval of a framework for carrying out a preagreed process when conditions appear that both sides have delivered the preagreed services. It's worth noting that smart contracts on the blockchain can go beyond simple activities and include more detailed instructions in their code. Applying certain rules that regulate a wide range of options [6, 7]:

1. Fact-based functionality: when triggered by external data that identify a specific and preagreed event (without them being primarily related to human intervention), smart contracts can modify other data.
2. Functionality based on external data: these data can be provided by reliable data sources that can provide dynamic, feedback information in smart contracts.
3. Functionality based on enforcement and proof: contracts may, based on the information provided, “enforce the functional application of a particular requirement and may demonstrate that certain conditions are met or not met.
4. Functionality based on changes. These capabilities involve monitoring changes in system status over time and adapting to them.

In this paper, a blockchain-based verifiable user data access control policy for secured big data storage in the cloud is proposed based on the design of a data exchange network between systems that use cloud computing utilizing blockchain technology. The systems will be able to transmit securely, control, and detect data while sharing medical data with other medical institutions and research institutes without any risk to their privacy. The method includes utilizing blockchain components to distinguish the suspicious behavior successfully and repudiate access with the implementation of the model. The aim is to produce a cutting-edge system for applying classified access policies to secure cloud resources powered and enhanced by blockchain technology.

## 2. Literature Review

The use of the blockchain technology is relative concept in the research community. However, researchers have focused on the utilization of the most aspects of this innovative technology, and one of the most promising areas of research is the combination of the access control mechanisms with the blockchain. Chinnasamy et al. [8] in 2017 presented for the first time a distributed access control framework by combining blockchain with an access control model. They introduced smart contracts as a way to implement contextual access control restrictions and make authorization decisions. They also used blockchain to enforce access policies in dispersed situations where there is no central authority and to ensure that policies are enforced correctly and uniformly.

Also, Macías and Guitart [9] proposed using blockchain technology as an access control tool for representing and transferring resource access rights from one user to another. They advocated storing the representation of these rights in the form of transactions on the blockchain. They also employed attribute-based access control (ABAC) policies, which combine a collection of rules expressing conditions over a set of attributes associated with the subject, resource, or environment. In addition, Uchibeke et al. [10] in 2018 implemented identity-based access control (IBAC) and role-based access control (RBAC) on the Hyperledger Fabric blockchain, a private and permissioned scheme led by IBM, to achieve access control methods for big data (RBAC).

They built the request, grant, revoke, verify access, and view asset actions for each access control model. Finally, they contrasted the outcomes of both implementations and discussed the stability difficulties caused by the Hyperledger Fabric blockchain's newness. Finally, Rouhani and Deters [3] gave an outline of the current access control techniques' difficulties and how the blockchain can assist overcome them. They also looked at the obstacles that come with adopting a blockchain-based access control system as well as presenting an overview of related research projects and categorizing them based on different domains and access control methods.

On the other hand, Ghaffari et al. [11] conducted a comprehensive study to provide a comprehensive picture of the current state of the art in integrating blockchain and smart contracts in access control and authentication techniques. They began by outlining the history of distributed ledger technology, proposing a taxonomy for categorizing current methods based on type, application environment, and blockchain exploitation. They also looked at existing blockchain-based authentication and access control mechanisms in a variety of settings, including health care. Algarni et al. [12] suggested a solution based on a multiagent system and a blockchain to handle the delivery of lightweight and decentralized secure access control of an IoT system. The fundamental goal of this strategy was to create blockchain managers (BCMs) to secure IoT access control and allow secure communication between local IoT devices. Dar et al. [13] in 2021 attempted to give an analysis of the available empirical evidence by attempting to synthesize the literature in order to comprehend the state of the art in blockchain-based access control methods for underlying platforms. They found a sufficient number of relevant primary research and focused on many topics such as single point of failure, security, and privacy.

They also conducted a meta-analysis and thematic synthesis on the utilization of various blockchain platforms, application domains, and blockchain features. Gao et al. [14] proposed a blockchain-based security sharing mechanism for personal data as a solution to this challenge. They combined four independent components: the blockchain, ciphertext policy, attribute-based encryption (CP-ABE), and the interplanetary file system (IPFS). To maximize the scheme's decentralization, this is a user-centric scheme in which the data owner encrypts the sharing data and saves it on IPFS.

Most of the above literature is utilizing the blockchain technology but rarely evaluate their work against certain cyberattacks. In the present work, we not only propose a novel scheme for a specific sector like health care but we also compare it against specific threats.

## 3. The Proposed System

To achieve the high demands on big data storage, the cloud computing mechanism offers a solution because it provides controlled and flexible data processing and exchange mechanisms as well as their respective storage spaces [15]. The increased interest has expanded in the field of health, including medical and research institutions and their cooperation. But despite the advantages that cloud computing offers, it lacks the functionality associated with data exchange due to the risks involved in exposing its content. For data proprietors, there's a risk that the data collected will end in the hands of malevolent users. In this context, the fear of violating the regulations and the exploitation of data creates an atmosphere of mistrust that does not ensure the implementation of data exchange. Blockchain technology can offer the right solution to deal with this problem through its attractive properties such as its decentralized and unchanging nature [9, 16].

### 3.1. Basic Functions of the System

The model proposed and described is based on the blockchain mechanism and specifically on the properties of smart contracts, but also cloud computing, and is used to exchange medical records between service providers, providing data control and at the same time proper management of their large volume. The actions of the beneficiaries are constantly monitored with the contribution of various mechanisms, and the violations are treated.

#### 3.1.1. Blockchain Network

The pieces of information are stored in the blockchain. The requests that the system receives from external users for access to the desired data are created into blocks and are later transmitted to the chain during the delivery of the package to the user. The last action completes the creation of the block and allows its transmission to the blockchain network. Each block is identified by its unique value which is also its identity. The significance of executing side blocks in the network is to preserve an effective log to investigate violations of terms [17].

They are attached to parent blocks and include indexed references, identical to those listed in the smart contracts database. Creating multiple network connections brings together a complete collection of reports. A block is created from a processed form, which represents a request received from an external user and contains information related to the receipt of the request, the processing, and delivery of the data.

A peer-to-peer network is outlined on the concept of peers who work at the same time as clients and servers to the other hubs of the arrangement. The foremost common application of peer-to-peer organization is the distributed hash table (DHT) [16], which employs a hash function to certify ownership to the organization of nodes [18]. This allows peers to find resources employing a hash table: the records are stored in DHT in pairs [key, value], and each node can recover the value related to a given key.

A DHT is a sophisticated decentralized framework that gives an effective research mechanism in which any participant node can recover the value related to a given key. Each node needs to be coordinated with only a small part of the total system nodes—usually *O* (log *n*) where *n* is the system nodes—so that it needs to be a small amount of work for each change in the participating nodes (e.g., withdrawal). There are some classic issues that DHTs must deal with, such as load balancing, data integrity, and performance.

Nodes and keys receive m-bit IDs, for which the basic hash function is the SHA-256 algorithm, and consistent hashing is essential for chord robustness and high performance. According to the chord search protocol, nodes and keys are arranged in a circle of identifiers containing 2*m* positions, with values from 0 to 2*m* − 1 (the *m* should be large to avoid collisions). Each node has a successor and a predecessor.

The successor to a node is the next one in the clock cycle. Respectively, its predecessor is the immediately preceding one (at the same direction of rotation). If there is a node for each possible ID, then node 0 is the successor to node 1 and its predecessor is node 2*m* − 1. Of course, usually, there are “gaps” in the sequences of nodes.

For example, the successor of node 159 can be node 200 (there are no nodes with IDs between 159 and 200), which means that node 200 has a predecessor the node 159 [19, 20].

When a new node is entered, three properties must be retained [16, 21]:

1. The successor of each node must point correctly to the next one
2. Each key *k* must be stored by the successor (*k*)

The finger table of each node must be correct.

Every network transaction has one or more inputs and outputs, all of which are recorded on the blockchain. These outputs create chunks, which are recognized by the whole network and made available to the owner for future transactions. In addition, each input/output has a time-stamped function associated with it.

The hash outputs of transactions are used to uniquely identify them, whereas the output index of specific transactions is used to identify them.  Figure 1 depicts an example of this technique.

Network's proof of work takes advantage of the seemingly random nature of cryptographic hashes. A party must construct a hash of the block header that does not exceed a particular value in order to establish that it did a given amount of computational labor to create a block. The hashing technique used is double SHA-256, and the specified structure is a hash that is less than or equal to a target value *T*. The purpose is to find a hash that is numerically less than the target, which we name the value threshold target. We alter a variable called nonce every time we want to change the hash result, usually by incrementing it by one. The likelihood of finding a nonce *n* for a given message (msg) such that *H* = SHA2562(msg||*n*) is less than or equal to the target *T* is [16, 20]

(1) $$\begin{array}{c} P\left[H\leq T\right]=\frac{T}{2^{256}}. \end{array}$$

The following quantity of computations is the average number of tries completed by a party attempting to find a proof of work:

(2) $$\begin{array}{c} T\left[H\leq T\right]=\frac{1}{P\left[H\leq T\right]}\\ =\frac{2^{256}}{T}. \end{array}$$

Finally, by simply assessing the nonce that comes with the message, it is simple and quick to determine whether it is genuine proof of work:

(3) $$\begin{array}{c} \text{SHA}256^{2}\left(\text{msg}\left\|\;\right.n\right)\leq T. \end{array}$$

#### 3.1.2. Cryptographic Keys

Encryption keys [5, 22, 23] are labeled to perform specific tasks related to their security on the system. For the exchange and transmission of data between “unreliable” nodes, encryption keys are required, ensuring a level of security in the system. Specifically, the user's private key that sends the request for access to the system creates its private key and uses it to put its own “digital signature” on it. Respectively, the public-key of the user sends it in combination with the request, the public-key that he has created to be used for the verification of his identity through the control of the digital signature. The smart contract key is also a pair of keys generated by the authenticator which are attached to the smart contract delivered to the user so that he can decrypt the data he received but at the same time follow the rules of the smart contract so that there is control over the use of data by the system [24, 25].

The following is the mathematical formula for deriving public-key cryptography, with *C* denoting the encrypted message:

(4) $$\begin{array}{c} C=\text{encrypt}\left(M,K\text{pub}\right),\\ M=\text{decrypt}\left(C,K\text{pri}\right). \end{array}$$

The suggested method's public-key cryptography is based on elliptic curve multiplication. The following function, which produces an elliptic curve, is used to define the curve:

(5) $$\begin{array}{c} y^{2}=\left(x^{3}+7\right)\mathrm{mod}p. \end{array}$$

In summary, a user who wants to access file sets from the system and the data holder creates a pair of private and public-keys. Upon receiving, the data holder confirms the validity of the request and the identity of the user, verifying the public-key signature of the user. The results obtained from the retrieval of the requested files are processed by the system, and then, before the file is delivered to the user, it is encrypted with a “contract key,” which is attached to the smart contract that is sent along with the data. By decrypting the file, the data holder gains full control over the actions performed by the user, as the smart contract is automatically activated [1, 24, 26].

#### 3.1.3. Triggers

The main role of the application of triggers is to allow smart contracts to indirectly connect the system with the external environment of the system since the latter cannot interact directly with structures outside the network [27]. They do not hold any information and only act as intermediaries for the smooth communication of the level of requests with the level of processing them. Triggers also update process statements to and from the level of requests based on smart contract features.

### 3.2. System Design

The design of the system is based on open architecture systems, where there is the independence that ensures the smooth cooperation and operation between the individual operating applications and subsystems of the information system and the network cooperation between applications and/or systems located in different computer systems. Its modular architecture also allows for future extensions and replacements, integrations, upgrades, or changes to discrete software or hardware components. Finally, the *n*-tier architecture allows the flexibility of cost and load distribution between central systems and workstations for the efficient operation of the network and the ease of its scalability.

#### 3.2.1. Users

They are all users whose intention is to access medical data, either for clinical or research purposes (e.g., health-care organizations, hospitals, research institutes, universities, and research scientists). Users send requests to the system for access to the data, which are subjected to a processing process.

#### 3.2.2. Request Receipt Field

The model consists of structures that receive, process, and respond to requests placed in the system and related to access to existing data. This level interacts directly with the data processing and transmission level and has built-in mechanisms to interpret and translate actions between the internal and external environment. In addition, users communicate directly with this mechanism to send requests. Its structural elements are [2] as follows:

1. Request conversion structure: it is responsible for converting requests into a format that can be recognized by the data processing and transmission field. The conversion results in a value that replaces the request and can be read by the system to retrieve the requested information. His final role is to respond and send a “response” to the applicant based on the request he has made.
2. Structure of “translation” of smart contracts [8, 28]: this system has the responsibility to translate the actions of smart contracts to and from their environment as it cannot operate outside a blockchain network autonomously.

#### 3.2.3. Data Processing and Transmission

The model includes components that assist the user's request for data access. Additionally, calculations are performed on the requested data, and functions are added which detect any action. Algorithmic processes are applied to the data and undertake to report on the actions performed. The results of each action that has been completed are transmitted to an unchanged network that guarantees fair control.

The system is also responsible for authenticating any request and action regarding access to digital medical records. Existing level entities are authenticator, nodes of processing and consent, smart contracts production structure, smart contract database, and blockchain network [2, 6, 29].

#### 3.2.4. Cloud Computing Database

The database contains functions that are used to perform specific tasks. Only authorized personnel from the consent nodes have access to this system, as they host private information that requires safe methodologies adequately to ensure high-level protection. To access the data in this database, the required information is transmitted through calculations so that it can be shared [1, 30].

### 3.3. System Functionality

The operation of the individual applications, subsystems, and solutions consisting of the distinct parts of the information system ensure that the greatest possible uniformity is achieved in the interfaces between the different subsystems and in the way they operate, and common and friendly presentation modes will be chosen in terms of user interfaces, with applications and system scalability to be ensured. Also, the use of flexible management systems allows the functional control of the large volume of data, the increased availability of the system, and the possibility of controlling access to the data [3, 21].

#### 3.3.1. Reception of the Request

The user sends a request to access specific data. The request is digitally signed by the user via his previously created private key. The request initially meets the level of receipt of requests. The triggers in the system convert the request into a structure that can be read by the system that processes and transmits the data and transmit it to that level. Initially, the authenticator verifies the legality of the request by checking the signature, using the corresponding public-key of the applicant which has been distributed by the user when sending his request [17]. The process proceeds further if there is a valid signature, otherwise interrupted, and considered as an invalid request.

#### 3.3.2. Request Processing

Once the request is approved, the processing and consent nodes undertake to convert it into a suitable form which will include, in addition to the desired data, a unique value representing the identity of the applicant (user ID) but also a time stamp of the time of receipt of the request. The two values are attached to the form, after first being hashed, through a mathematical hash function. The reason for which the specific data are requested is also indicated in the form, and finally, it is transferred to the existing database.

This database takes the form, retrieves the requested data, and sends it back to the processing and source level where the first modification by the consent nodes will occur. The time stamp of the request created on the form will be noted in the retrieved information. Consent nodes then send a request to the center of smart contracts to establish rules about the requested data [6, 7]. The corresponding smart contract will be generated and integrated into the form along with the data.

#### 3.3.3. Distribution of the Requested Data

The new form that is the result of the previous processing is sent to the authenticator to undergo through the final stage. The authenticator generates an encryption key and points it to the smart contract that has been created. With the key, the user will be able to decrypt the requested data. This is important to ensure the secure transmission and detection of information. At the same time, the consent nodes construct a chain of block-based piece of data requested by the user and transmit it to the blockchain according to the chronological order in which it is created. As expected, the block will have a unique identifying value, following the cryptographic methods it has been subjected to, following the blockchain network way of operation.

The packet that has been created by processing the requested data retrieved from the existing database includes the data, the value of their “identity” (data ID), and the smart contract with the terms of use of the data. Eventually, the entire packet is encrypted by the authenticator so that it can only be identified by the holder of the appropriate private key, and by entering the user ID, it is sent back to the request system from where it was initiated [1, 30]. The smart contract is the reason for the effective monitoring of the package.

#### 3.3.4. Delivery of the Data to the User

The user receives the edited packet and decrypts it with his private key. His security must somehow be validated. At this point, the contracts that have been configured by the processing system will play a key role. With the key attached to the smart contract, the user decrypts the data, and it is automatically activated. Any action on the decrypted data received by the user is reported and sent to the level of receipt of requests, from where it is translated and transferred to the level of processing and specifically to the consent nodes. They, in turn, store the reference in the blockchain chain to a side block that is inextricably linked to the block added during the previous procedure.

The reason for keeping the file containing the actions performed in the data is to prevent their malicious use. The installation of such reports reflects the ability of the smart contract to activate specific conditions when performing any transaction that is directly related to the requested data [31, 32]. Through this property, the control of the documents available to the user is achieved.

#### 3.3.5. The Function of Smart Contracts

Smart contracts operate as systems that execute predefined instructions when performing actions that follow an organized framework. They are used to report actions related to the data requested by the user system and allow the data owners to secure and control them, as they will be monitored in a controlled environment, eliminating the relationship of trust required between the owner and the user. As mentioned above, reports about the actions of the data resulting from the user's system are updated and transmitted to the blockchain network. A set of actions can be applied to the data received by the user, which will activate the rule-based smart contracts. Data sensitivity can be categorized into high and low.

This is determined by the consent nodes when they obtain the data from the existing database. Based on the degree of importance of the package, some actions are excluded from the list of malicious acts, while others are violations [6, 28].

The identity of the data specified in the smart contracts gives an advantage in creating an effective medium so that the consent nodes can map, process, and verify the corresponding unique block. Comments are generated to describe the user-performed actions in the data. In most cases, they are comments of infringement or exclusion.

By extracting a key through specific commands, they are encrypted and stored in the smart contract database. The rights declared by the data holder are defined on the smart contracts. Unreliable data are handled appropriately by the owner [22, 26].

#### 3.3.6. Data Exchange between the Database and the Consent Nodes

The exchange of data is crucial for secure operation of the information-sharing between entities where there is no trust. The data output from the database must maintain the integrity, and for this reason, their exchange methods need to be designed and structured with great care. For the approved request, the database makes a copy of the data and forwards it to the consent nodes which are responsible for configuring the entire package. The package includes, in addition to the data, an identifier of these (data ID) but also an identifier of the consent node that undertook the processing. The node in charge of the modification verifies the data received by comparing its type with the requested request. They are classified on a scale characterized by high or low sensitivity. For a highly sensitive data set, there is a need for greater security and anonymity.

The actions performed using the sent information are recorded in a format that will eventually convert them into blocks and will be added to the network. The result is obtained from the data management node by node. Once this is considered accurate, they are returned to the first node. The consent node sends a request stating the level of data sensitivity to the smart contract generator to generate the corresponding contract with the rules.

Eventually, it is attached with the requested data and the completed file is encrypted by the authenticator with the user's public-key, and a time stamp is issued at the end of the process. All processing times are recorded by the consent node to allow efficiency-based optimization. In addition, the form with the performed actions includes the contribution of the second node [1]. The file is formatted in blocks and is now ready to be added to the blockchain system.

#### 3.3.7. Main Block Structure in the Blockchain Chain

Each block, as mentioned in the description of blockchain technology, is uniquely identified and described by a fragmented value that has been calculated. The block includes its size as well as the block header. The blockchain uses SHA-256 to generate the hash value of a message *M*. The result of the SHA-256 is a 256-bit message summary [16, 21].

The header has gone through the fragmentation process through the SHA-256 algorithm and plays an important role in the blockchain, making it unchanged. It contains the fragmented value of the previous block that was added to the chain, so any change to a block should change the entire chain starting with the original block, the genesis block.

This fact ensures the integrity of the network since there is a maximum guarantee that it is not possible to achieve this goal. The mechanism also guarantees the origin of the data, so in case of malicious activity, the mismatch of the blocks will warn the system to enable accurate data verification. The block header consists of the rules to be followed for data validation in the block and the properties that will have [25].

In addition to the fragmented value of the previous block contained in the header, part of it is the Merkle tree root, which contributes to the security of the chain by ensuring that none of the blocks can be modified without transforming the header. The Merkle tree root results from the hashing of all records received by the block. The output is the result of the SHA-256 algorithm as used throughout the header. An important part of the heading is the time stamp of the creation of the block and a nonce value, which is a random number set by the consent nodes to generate the fragmented header value in conjunction with the target difficulty value [33].

The block contains an activity counter, the function of which is to log the amount of malicious attempts concerning the data recorded in it by time stamps, and data section. The time stamps are classified based on the time of receipt of the request, the time required for its processing, and the time needed to send the file to the user. The data section consists of the identity of the data owner, their sensitivity, the purpose of the request, the identity, and the signature of the processing and consent node. The arrangement that defines the whole block structure is the locking time [34].

#### 3.3.8. Side-Block Structure

A side block is a form that comes from attaching a section to a master block, producing a new block with its own identity. The block side consists of its size but also the header with the sections found in the main block, in particular, the version of the block that uniquely identifies the references used to create it, the fragmented value of the previous block, the Merkle tree [18, 35] root of all records, its time stamp creation, the target difficulty value, and the nonce value. The listed components have the similar properties as the parent blocks but are attached to the side blocks. Like the parent block, the side block also has a counter for malicious activity, which is recorded in a report. It not only consists of the time stamp of the action, the action itself, the identity of the data holder, and the identity of the user but also the identity and signature of the consent node. The block is “locked” in time and attached to the parent block of the blockchain. Traces of data and reference can now be traced.

#### 3.3.9. Overlay Layer

This is an extra layer that was included in the blockchain stack layer to map the communication arrangement between the participants. Overlay nodes are an abstract logical path and can be thought of as associated with virtual links, each of which underlies the physical network topology. [22, 23].

#### 3.3.10. API Layer

It is the application programming interface that allows external applications or users to interface with the blockchain. It allows the extraction of information from one system to another in a clear way.

The proposed blockchain-based verifiable user data access control policy mechanism is depicted in Figure 2.

## 4. Attacks Scenario

The scenario under consideration will focus on questions of finding closest neighbors and will demonstrate that the proposed system supports the secure processing of such questions under different intruder capabilities [36]. The *k*-nearest neighbors (k-NN) method is a critical parsing function of common data processing operations (e.g., classification or grouping) [24, 37].  Figure 3 shows the model for secure computing of encrypted databases [24].

In this model, the owner (user_1) of a database needs to execute some DB queries. To take advantage of a service provider's computing resources, it exports the database to an encrypted scheme (encrypted DBMS). Therefore, all blocks are encrypted by user_1 in order to proceed further to the encrypted DBMS. On the encrypted DBMS *E*(DB), all submitted queries by any user are also encrypted, resulting in an encrypted response *R* (e.g., *R* is an encrypted set of blocks of the answer to a k-NN query) [25, 38, 39]. All users must agree on a specific encryption system that ensures the integrity of the whole system. The proposed encryption model consists of the following elements: a secret key *K*, an ET() database encryption function, a set of Aux auxiliary operators, and a decryption function *D*() as a result [36].

In particular, the proposed encryption scheme requires that the encrypted queries and DB points should be encrypted differently ([ET() ≠ EQ()]). The graduated product of *p* and *q* (represented by the column vectors) can be represented as *p*^T^*Iq*, where *p*^T^ is the inverse of *p* and *I* is an identity register *d* × *d*. I can be replaced by MM^−1^ for any reversible register *M*, i.e., *p*^T^*q* = (*p*^T^*α*) (*M*^−1^*q*). If we set *p*′ = *E*_T_(*p*, *K*) = M_T_*p* and, respectively, *q*′ = EQ(*q*, *K*) = *M*^−1^*q*), it is not possible for one to determine the value of *p* or *q*, respectively, from *p*′ or *q*′ without knowing *M*. Also, *p*′^T^*q*′ = *p*^T^MM^−1^*q* = *p*^T^*q*, i.e., the graduated product of type 2 is retained. If *p*′1 and *p*′2 are the encrypted points of *p*1 and *p*2 in DB, respectively, then *p*′1^T^ p2′ = *p*1^T^ MM^T^ p2, which is not equal to p1^T^p2 in general. Therefore, type 1 and 3 grade products are not retained. Thus, we can perform ASPE using *M* and *M*^−1^ as transformations function of DB points and queries, separately. Also, *p*′^T^*q*′ = p^T^MM^−1^*q* = *p*^T^*q*, i.e., the grade 2 product is retained [24].

### 4.1. Attack Models

In the model, we assume that the encrypted DBMS, which may be in a third party (e.g., cloud service provider), is not secure. Therefore, we assume that an intruder (user_3-attacker) sees the encrypted DBMS environment [22, 25, 40]. Specifically, the attacker has access to the encrypted DBMS (encrypted queries, results, etc.) and in all components of the encryption system except from key (ET(), EQ(), *D*()), Aux, etc.).

We assume that the attacker's goal is to retrieve a portion of the DBA ⊆ DB database and that he can perform cryptanalysis algorithms relative to the size of the encrypted database. In computational complexity theory, *P*, (nO(1)), is a fundamental order of complexity that contains all decision problems that can be solved by a deterministic turing machine in polynomial time. Our goal is to prevent the attacker from gaining part of the database. In addition to *E*(DB), the attacker may have additional information about the original data. To evaluate the encryption system, we will classify the attackers at different levels based on the knowledge they possess. Specifically, Level 1, the attacker only observes the encrypted database *E*(DB). Level 2, the attacker knows a set of simple blocks P in DB but does not know the corresponding encrypted values of these blocks in *E*(DB). Level 3, the attacker observes a set of P blocks in DB and knows the corresponding encrypted values of these blocks.

Among the three attack levels defined, we observe that level 2 attacks describe practical scenarios. This is because in some applications, it is not difficult to observe a small number of simple database blocks (e.g., by artificially inserting “spy” blocks into the database). In addition, it is considered that the attacker cannot observe the simple questions in all cases. In particular, the attacker is not allowed to pretend to be user_2 and query the database. Note that level 3 attacks are rare in practice, as it is not easy for someone who does not have the encryption key to associate known simple blocks with their encrypted values.

### 4.2. Queries of k-NN Neighbors in the Model

We will focus on questions from nearest k-NN neighbors and explain how the proposed encryption scheme (which includes the above five components) responds to the secure support of k-NN applications in the model. A k-NN query looks for *k* points in a database that are closest to a given query point *q*. Note that each database set can be modified as a multidimensional point if we consider some of its features as dimensions and their values as coordinates. One approach to securely supporting k-NN is the distance preserving transformation (DTP) for point encryption so that the distance between any two encrypted points in *E*(DB) is the same as that between the corresponding DB starting points. Given this property, k-NN can be computed in the encrypted database. Unfortunately, this transformation is proving to be unsafe in practice. If an attacker has access to the encrypted DPT database *E*(DB) and knows a few points in the plaintext DB database, he can fully recover the DB.

Similar k-NN query computing problems on an unreliable platform are studied services where users query an unreliable server that maintains the data. These applications focus on protecting users' privacy (query content) since the database is considered to belong to the server. While some studies also concern the privacy of files in the database, k-anonymity is adopted as a standard for database protection. We observe that k-anonymity has a different security goal compared to the proposed model. K-anonymity aims to prevent an attacker from locating a person from the database, but the contents of the database may be exposed. In addition, most of these models require the existence of a trusted intermediate (anonymous location) that handles the transformation of data and queries. This piece, in addition to being a single point of attack, undermines performance as every question and result must go through it.

### 4.3. Distant Recovery Encryption

In the k-NN calculation, the distances between the database points at a query point are calculated to find the nearest neighbors to the search point, so an encryption scheme that allows the system to calculate *d*(*p*1, *p*2) at *E*(DB) for base points *p*1 and *p*2 at DB is not safe. However, the proposed encryption system is secure against level 2 attacks, as it does not allow distance calculation.

*Distant Recovery Encryption (DRE)*. We have an *E*(*p*, *K*) which is the encrypted value of a point *p* in DB. *E* is recoverable from a distance if and only if there is a computational procedure *f* for which for every *p*_1_, *p*_2_*K*, *f*(*E*(*p*_1_, *K*), it holds that *E*(*p*_2_, *K*)) = *d*(*p*_1_, *p*_2_). If *E* is DPT, we have *d*(*E*(*p*_1_, *K*), *E*(*p*_2_, *K*)) = *d* (*p*_1_, *p*_2_). For a point *p* in DB represented as a column vector, the encrypted value *E*(*p*, *K*) of *p* of a DPT *E* can be expressed as Np + *t*, where *N* is a rectangular register *d* × *d* and *t* is a two-dimensional column vector. The distance between the points is maintained, that is, *D* (*p*_1_, *p*_2_) = *d* (*E* (*p*_1_, Κ), *E* (*p*_2_, Κ)). Therefore, DPT supports efficient k-NN calculations. However, DRE and therefore DPT are secure and resilient in the proposed scheme.

Specifically, and assuming that a DRE *E* is used to encrypt the DB to get the *E*(DB), a level 3 attacker with *H*=〈*E*(DB), *P*, *I*〉 can retrieve DB if P contains at least *d* + 1 points *x*_*i*_ (1 ≤ *i* ≤ *d* + 1) so that the set of vectors {*x*_*j*_ − *x*_1_ | 2 ≤ *j* ≤ *d* + 1} is linearly independent. Therefore, although no DRE can survive this level 3 attack, this pattern survives as DHT uses a hash function to assign file ownership to network nodes which generate a 256-bit key *k*. Specifically, the proposed system uses an encryption function that does not reveal distance information as data of two points *p*1, *p*2 in DB, and it must be decided which of the two points is closest to a question point *q*, as well as

(6) $$\begin{array}{c} \sqrt{{\left\|p1\right\|}^{2}-2p1*q+{\left\|q\right\|}^{2}}\geq \sqrt{{\left\|p2\right\|}^{2}-2p2*q+{\left\|q\right\|}^{2}}, \end{array}$$

where ||*p*|| represents the Euclidean norm of *p* and *∗* represents the gradient system. ||*p*||2 can be represented by *p∗p*. Thus, inequality is subdivided into several calculations of gradients. This indicates a graded encryption of Espe product conservation, i.e., ∀*p*1, *p*2 ∈ B, *p*1 *∗p*2 = Espe (*p*1, *K*) *∗* Espe (*p*2, *K*), to calculate k-NN.

Even if the attacker manages to “upgrade” the knowledge of level 2 to level 3 using the “signature linking” attack, the proposed scheme is a guarantee and in particular, if at level 2, *H*=〈*E*(DB), *P*〉, the intruder constructs the signature of P from the distances per pair between every two points in *P*. Suppose the points in *P* are classified and *P* = {*x*_1_, *x*_2_,…, *x*_|*P*|_}. The signature of *P*, sig (*P*), is a vector of size |*P*|*C*_2_ whose form is (*d*(*x*_1_, *x*_2_), *d*(*x*_1_, *x*_3_),…, *d*(*x*_1_, *x*_|*P*|_), *d*(*x*_|*P*|_−1, *x*_|*P*|_)). The attacker tries to find a sorted set of encrypted points *Q* in *E* (DB) so that |*Q*| = |*P*| and *Q* give the same signature as *P*. Let *Q* = {*x*_1_′, *x*_2_′,…*x*_|*P*|_′}. Sig (*Q*) is (*f* (*x*_1_′, *x*_2_′), *f* (*x*_1_′, *x*_3_′),…, *f*(*x*_1_′, *x*_|*P*|_′)), *f*(*x*_|*P*|_′ − 1, *x*_|*P*|_′)). If there is only one set *Q* with that signature, the attacker can conclude that *x*_*i*_′ is the encrypted *I*(*x*_*i*_) = *x*_*i*_′ for all *x*_*i*_∈*P*. With this *I*, *H*=〈*E*(DB), *P*, *I*〉, and the attacker can carry out a level 3 attack. The success of the signature linking attack is based on two issues: if *Q* is simple to discover and in case is conceivable that another set *Q*′ gives the same signature collision.

For the first question, we notice that the search space in the proposed shape is huge and cannot be effectively reduced by the “pruning” technique. For the second, we are able to appear that the likelihood of a signature conflict is extremely impossible. Moreover, indeed in case different *Qs* with the same signature as *P* are recognized, the attacker cannot increment the estimate of *P* to diminish the likelihood of a collision and rehash the attack as within the proposed design, the item maintenance encryption is not remotely retrievable which is given as follows:

(7) $$\begin{array}{c} f\left(p1^{\prime },p2^{\prime }\right)=\sqrt{p1^{\prime }*p1^{\prime }-2\left(p1^{\prime }*p2^{\prime }\right)+p2^{\prime }*p2^{\prime }}\neq d\left(p1^{\prime },p2^{\prime }\right). \end{array}$$

Therefore, the encryption function ET is not remotely retrievable as if the encryption *E* is remotely retrievable (i.e., *E* is DRE), then there is a computational procedure *f* such that for all points *p*_1_ and *p*_2_ and any encryption key *K*_1_, it holds that *a*1 = *E* (*p*_1_, *K*_1_) and *a*_2_ = *E* (*p*_2_, *K*_1_), and we have *f* (*a*_1_, *a*_2_) = *d* (*p*_1_, *p*_2_). That is, considering the encrypted values *a*_1_ and *a*_2_, the distance *d* (*p*_1_, *p*_2_) can be calculated from *f*, regardless of the encryption key.

## 5. Conclusions

The blockchain-based verifiable user data access control policy for secured big data storage in the cloud that was analyzed is based on the design of a data exchange network between systems that use cloud computing utilizing blockchain technology. The design includes the utilization of blockchain components to successfully distinguish the suspicious behavior and repudiate access with the implementation of the model, and the systems will be able to securely transmit, control, and detect data, while sharing medical data with other medical institutions and research institutes, without any risk to their privacy.

The variety of solutions offered and the costs involved are indicative of how difficult it is to secure a similar system in a hostile environment. It is reasonable to conclude that its securing requires specialized ways of assigning IDs to the nodes, dispersing the nodes, instant data copying, and an access mechanism that offers high possibilities of safeguarding security and privacy. In any case, despite the possibility of achieving a practically acceptable level of security in critical applications, it is obvious that a lot of research effort is still required as the requirements are high and constantly increasing.

## Figures and Tables

**Figure 1:** Transaction output reference computation.

**Figure 2:** Proposed blockchain-based verifiable user data access control policy.

**Figure 3:** The proposed attack scenario.

## Data Availability

Data are available on reasonable request to the author.
